# Chaperonin CCT-Mediated AIB1 Folding Promotes the Growth of ERα-Positive Breast Cancer Cells on Hard Substrates

**DOI:** 10.1371/journal.pone.0096085

**Published:** 2014-05-01

**Authors:** Li Chen, Ze Zhang, Juhui Qiu, Lingling Zhang, Xiangdong Luo, Jun Jang

**Affiliations:** 1 Breast Disease Center, Southwest Hospital, Third Military Medical University, Chongqing, China; 2 Burn Research Institute, Southwest Hospital, Third Military Medical University, Chongqing, China; 3 National Key Laboratory of Trauma and Burns, Chongqing Key Laboratory of Disease Proteomics, Chongqing, China; II Università di Napoli, Italy

## Abstract

Clinical observations have revealed a strong association between estrogen receptor alpha (ERα)-positive tumors and the development of bone metastases, however, the mechanism underlying this association remains unknown. We cultured MCF-7 (ERα-positive) on different rigidity substrates. Compared with cells grown on more rigid substrates (100 kPa), cells grown on soft substrates (10 kPa) exhibited reduced spreading ability, a lower ratio of cells in the S and G2/M cell cycle phases, and a decreased proliferation rate. Using stable isotope labeling by amino acids (SILAC), we further compared the whole proteome of MCF-7 cells grown on substrates of different rigidity (10 and 100 kPa), and found that the expression of eight members of chaperonin CCT increased by at least 2-fold in the harder substrate. CCT folding activity was increased in the hard substrate compared with the soft substrates. Amplified in breast cancer 1 (AIB1), was identified in CCT immunoprecipitates. CCT folding ability of AIB1 increased on 100-kPa substrate compared with 10- and 30-kPa substrates. Moreover, using mammalian two-hybrid protein-protein interaction assays, we found that the polyglutamine repeat sequence of the AIB1 protein was essential for interaction between CCTζ and AIB1. CCTζ-mediated AIB1 folding affects the cell area spreading, growth rate, and cell cycle. The expressions of the c-myc, cyclin D1, and PgR genes were higher on hard substrates than on soft substrate in both MCF-7 and T47D cells. ERα and AIB1 could up-regulate the mRNA and protein expression levels of the c-myc, cyclin D1, and PgR genes, and that 17 β-estradiol could enhance this effects. Conversely, 4-hydroxytamoxifen, could inhibit these effects. Taken together, our studies demonstrate that some ERα-positive breast cancer cells preferentially grow on more rigid substrates. CCT-mediated AIB1 folding appears to be involved in the rigidity response of breast cancer cells, which provides novel insight into the mechanisms of bone metastasis.

## Introduction

Bone metastases occur in more than 70% of breast cancer patients and lead to increased morbidity and mortality [1]. Clinical observations have indicated a strong association between estrogen receptor α (ERα)-positive tumors and the development of bone metastases [2]. In spite of its clinical importance, the underlying cellular and molecular mechanisms that drive bone metastasis remain elusive.

Paget proposed that breast cancer cells “seed” tissues of metastasis, “the soil,” and that each must contribute to the predictable frequency of organ-specific metastasis [3]. Human clinical data and genetic mouse models of breast cancer have indicated that ERα-positive tumor cells favor bone as the first site of distant metastasis [2], [4], [5]. The ER-positive status of breast tumors is associated with a higher rate of both relapse to the bone and late-onset bone metastasis [6], [7]. Patients with ER-positive breast cancer constitute a major clinical population who are at risk for bone metastasis [2]. Much progress has recently been made with respect to tumor cell-specific gene profiles that can predict organ-specific metastasis [4]; however, it is still unclear whether the bone harbors inherent biological characteristics that make secondary sites more attractive than others during ERα-positive breast cancer metastasis.

Several recent studies have shown that the rigidity of the substrate not only affects stem cell differentiation [8], but can also regulate other cellular outcomes including growth, motility, invasiveness [9], tissue morphogenesis [10], and gene expression [11]. Matrix rigidity regulates invasiveness, and cancer cell invasiveness has been reported to increase with the rigidity of the matrix in soft hydrogels [10], [12]. Bone is a unique microenvironment that differs from all other body tissues; in particular, it is more rigid than normal breast tissue. The rigidity of the bone matrix not only affects tumor growth, but also alters the tumor cell response to growth factors [11]. Thus, we hypothesized that bone rigidity is closely related to a high incidence of bone metastasis in ERα-positive breast cancer cases.

To test our hypothesis, in the present study, we cultured ERα-positive human breast cancer cells (MCF-7 and T47D) in substrates of different rigidity and observed changes in cellular functions including the growth rate, cell spreading area, and cell cycle. By using stable isotope labeling with amino acids (SILAC) screening, we investigated the differential expression of the whole proteome of ERα-positive breast cancer cells in response to the rigidity of the substrate. Our results showed that complex chaperonin containing t-complex (CCTs) proteins (CCT1–8) expressed at a higher level in more rigid substrates compared with soft substrates. We also investigated the mechanism by which the CCTs and ERα pathways regulate cellular biological functions on different rigidity substrates. Our observations suggest that variations in the rigidity of the microenvironment might play a role the preferential metastasis of cancer cells to bone.

## Materials and Methods

### Antibodies, cDNA Sequences, and Reagents

Mouse monoclonal antibodies against human CCTα, β, γ, δ, ε, ζ, η, θ, β-actin, AIB1, ubiquitin, and ERα, and goat anti-mouse secondary antibodies were purchased from Santa Cruz Biotechnology (Santa Cruz, CA, USA). The control mouse IgG1 was purchased from DAKO (Glostrup, Germany), and the CCT1-8 and ERα cDNA sequences were purchased from I.M.A.G.E. Consortium (Lawrence Livermore National Laboratory; Livermore, CA, USA). MG132 (the proteasome inhibitor) and all other reagents were purchased from Sigma (St. Louis, MO, USA).

### Cell Culture

The human MCF-7 and T47D breast cancer cell lines (American Type Culture Collection; Manassas, VA, USA) were maintained in modified minimal essential medium (MEM) supplemented with 10% fetal bovine serum (FBS), 2 mM l-glutamine, and 20 µg/mL gentamycin. Cell cultures were grown at 37°C in a humidified atmosphere of 5% CO_2_ in a Hereaus CO_2_ incubator. While seeding the cells on silicone substrates of different rigidity, a defined medium, containing Dulbecco’s modified Eagle’s medium (DMEM)/F12 supplemented with 1.0 mg/mL human albumin, 5.0 mg/L human transferrin, and 5.0 mg/L bovine insulin was added, and cells were maintained. During the experiments, cells were grown on the defined media.

### Selection of Substrate Rigidity and Polydimethylsiloxane (PDMS) Concentration

The substrate rigidity experiments were performed as described previously [13]. Briefly, the concentration of the curing agent and base were varied to control the elastic modulus of the silicone substrate, based on a procedure described by Goffin et al. [14]. The Young’s modulus (E_Y_) values selected to simulate substrate stiffness were: 10, 30, and 100 kPa. Silicone substrates were produced by mixing the PDMS curing agent and base at ratios of 1∶65, 1∶48, and 1∶25, which were left to stand for 6 h. Subsequently, the silicone substrates were placed in a drying oven at **60**°C for 2 days.

### Protein Extracts

To prepare protein extracts, cells were harvested and washed three times with phosphate-buffered saline (PBS) (Sigma) and pellets were resuspended in radioimmunoprecipitation assay (RIPA) lysis buffer (50 mM Tris, pH 7.6, 150 mM NaCl, 2 mM Na_3_PO_4_, 4 mM EDTA, 10 mM NaF, 10 mM sodium pyrophosphate, 1% Nonidet P-40, and 0.1% sodium deoxycholate). Cell suspensions were supplemented with protease inhibitor cocktail (Roche; Mannheim, Germany), incubated for 30 min on ice, and clarified by centrifugation for 15 min at 15,000×*g* at 4°C.

### Growth Curves Analysis

The cells were seeded in 24-well plates at a density of approximately 1–2×10^4^ cells per well. At each time point, cells were collected by trypsinization and centrifugation. The cells were counted by using a hemocytometer. All samples were prepared in quadruplicate and the entire experiment was repeated twice.

### Flow Cytometry

MCF-7 cells (100,000 cells per well) were seeded in 6-well plates containing different silicone substrates (E_Y_ = 10, 30, and 100 kPa). The cells were harvested and washed with PBS at different time points. The cell pellets were conserved with 75% alcohol, stored at 4°C, and then analyzed using a flow cytometer (Beckman Coulter; Miami, FL, USA).

### SILAC

SILAC-based mass spectrometry has been shown to be a powerful strategy for characterizing protein complexes and identifying specific interactions. MCF-7 cells were maintained in SILAC media. Heavy arginine (^13^C6) and lysine (^13^C6 ^15^N2) were added to DMEM ‘heavy’ bottles, which was used to incubate ‘heavy’ (H)-labeled cells, whereas light arginine (^12^C6) and lysine (^12^C6 ^14^N2) were added to ‘light’ DMEM, which was used to incubate ‘light’ (L)-labeled cells, as shown as Figure 1. Cells were divided into two populations (H and L), and incubated in their respective media for 6 doubling times, and until passage 6. Once labeled, H-labeled cells were grown on 100-kPa silicone substrates, and l-labeled cells were grown on 10-kPa silicone substrates. Prior to harvesting the cells, they were serum-deprived for 24 h, and subsequently, the cell lysates were collected and lysed as described above (Fig. 1). The experiment was repeated four times. In each set of labeling experiments, we identified 5011 proteins and quantified the molecular chaperone CCT/TRiC in the four cell-lysate experiments. We then restricted our analyses to the four cell lysate experiments.

**Figure 1:** A simple experimental strategy for SILAC-based proteomics. MCF-7 cells were cultured on soft silicone substrate (E_Y_ = 10 kPa) in protein Label Light media, and on hard silicone substrate (E_Y_ = 100 kPa) in protein Label Heavy media, respectively. Protein lysates were prepared and mixed at a 1∶1 ratio. Sample complexity was reduced prior to LC-MS/MS analysis by fractionation at the protein level through SDS-PAGE. The expression levels of selected proteins were validated by Western Blot analysis. E_Y_: the Young’s modulus.

### Identification and Quantification of Dysregulated Proteins

The simple liquid chromatography tandem mass spectrometry (LC-MS/MS) workflow is depicted in Figure 1. In the filtered results, 103 proteins were upregulated, 48 were downregulated, and 112 were unchanged. We identified the expression levels of CCT proteins on silicone substrates of different rigidity by Western Blot analysis. The CCTs identified (1–8, or α–θ) were involved in protein refolding, and the refolding activity of β-actin was investigated.

### Immunoprecipitation

Eight micrograms of monoclonal antibody anti-CCTη, anti-CCTζ, or control mouse IgG1 were absorbed, respectively, on 35 µL of protein A/G sepharose (GE Healthcare) for 2 h at 4°C on a tube rotator. The pre-absorbed antibodies were then incubated with 200 µg of SaOS-2 or MCF-7 protein extract for 4 h at 4°C, then washed three times with RIPA buffer, and finally eluted with 20 µL of sodium dodecyl sulfate (SDS) sample buffer. Proteins were separated by 10% SDS-polyacrylamide gel electrophoresis (PAGE) and then electroblotted on a Hybond-ECL membrane (GE Healthcare) for 1 h at 4°C at 100 V. The membrane was saturated with 5% non-fat dry milk (BioRad; Hercules, CA, USA) for 1 h at room temperature and then incubated with anti-AIB1, Anti-ERα, anti-CCTα, anti-CCTη, or anti-CCTζ antibody at 4°C overnight. The secondary antibody conjugated with horseradish peroxidase (Amersham Biosciences; Uppsala, Sweden). Membranes were incubated for 1 min in Western Lightning Chemiluminescence Reagent Plus (Perkin Elmer; Boston, MA, USA) and the Western Blot signal was exposed and developed.

### Plasmids Construction and Bacterial Expression

The human full-length cDNA encoding the β-actin (GenBank accession no. NM_001101) protein was provided from I.M.A.G.E., and the human full-length cDNA encoding the amplified in breast cancer 1 (AIB1) (GenBank accession no. NM_006534) protein was amplified by polymerase chain reaction (PCR) from MCF-7 cells. Both full-length cDNAs were cloned in the pET 30a (+) expression vector (Novagen; Darmstadt, Germany) using *Nco*I/*Xho*I restriction sites, and were checked by sequencing. The expression of the resulting 6×His-fused proteins was induced with 0.4 mM isopropyl β-d-1-thiogalactopyranoside (IPTG) in *E. coli* BL21 (DE3). Bacterial cells were harvested by centrifugation for 15 min at 5000×*g* at 4°C; cell pellets were resuspended in lysis buffer (1 mM PMSF, 20 mM sodium phosphate, pH 7.4, 0.5 M sodium chloride, 5 mM imidazole), lysed by sonication, and clarified by centrifugation at 10,000×*g* for 30 min at 4°C.

The recombinant proteins were purified by IMAC affinity chromatography on a HisTrap HP column (GE Healthcare; Chalfont St. Giles, UK) connected to an Akta Purifier system (GE Healthcare). Lysates were loaded on a HisTrap column equilibrated in buffer A (20 mM sodium phosphate, pH 7.4, 0.5 M sodium chloride, 5 mM imidazole), and, after extensive washing, the His-tagged proteins were eluted with a linear gradient from 0 to 100% buffer B (20 mM sodium phosphate, pH 7.4, 0.5 M sodium chloride, 500 mM imidazole) in 20 column volumes. Collected fractions were analyzed by 12% SDS-PAGE.

### Folding Activity Assay

[^35^S]-labeled unfolded β-actin or AIB1 target protein was generated by expression in *E. coli* and purified as described by Gao et al. [15]. The refolding activities of cell extracts from MCF-7 and T47D cells were assayed and analyzed following dilution from denaturants of radiolabeled β-actin or AIB1 ∼500 ng into cell extracts, rabbit reticulocyte lysate (RRL) and human non-cancer liver (HNCL), diluted in folding buffer (80 mM MES/KOH, pH 6.8, 1 mM MgC_l2_, 1 mM dithiothreitol (DTT), 1 mM ethylene glycol tetraacetic acid (EGTA), 1 mM ATP). The protein concentration within the extracts was 12 mg/mL or 5 mg/mL. The reaction products were resolved on 6% non-denaturing polyacrylamide gels. The gels were then dried and exposed to a storage phosphor screen (Molecular Dynamics; Sunnyvale, CA, USA) and developed on a Storm PhosphorImager (Molecular Dynamics). All experiments were performed twice.

### Immuno-depletion of Cell Extracts

MCF-7 cell extracts on 100-kPa silicone substrates were immuno-depleted either using anti-ERα, anti-prefoldin (PFD) or anti-CCTζ antibodies. The extracts were incubated for 2 h at 4°C under gentle motion with the adequate antibody, and the protein antibody complexes were sedimented after overnight incubation at 4°C with Protein A Sephrose CL-4B beads (GE Healthcare) equilibrated in 50 mM Tris-HCl, pH 7.0. The supernatants were recovered, the protein concentrations were measured, and the ability of the immuno-depleted extract to refold [^35^S]-labeled unfolded AIB1 was assayed *in vitro*.

### Western Blot

Cells were lysed using RIPA buffer containing Complete Mini EDTA-free protease inhibitors (Roche; Branchburg, NJ, USA). The protein concentration was measured using the Bradford protein assay (BioRad; Hercules, CA, USA). For Western immunoblot, 30 µg of crude proteins was fractionized by SDS-PAGE and transferred onto nitrocellulose membranes. Membranes were blocked overnight at 4°C with 5% milk/PBS-Tween (w/v), and then incubated with primary antibodies for 1 h at room temperature. Membranes were then incubated for 1 h at room temperature with horseradish peroxidase-conjugated secondary antibodies (Amersham Biosciences). Membranes were incubated for 1 min in Western Lightning Chemiluminescence Reagent Plus (Perkin Elmer) and the Western Blot signal was exposed and developed. GAPDH was used as a loading control.

### Mammalian Two-hybrid Protein-protein Interaction Assays

The mammalian two-hybrid protein-protein interaction assay was performed as previously described [16]. Briefly, the full-length cDNA sequences of human CCT1–8 were amplified by PCR from cDNA sequences from I.M.A.G.E. and the DNA primers for reverse transcription (RT)-PCR were chosen based on GenBank accession numbers NM_030752 (CCT1), NM_006431 (CCT2), NM_005998 (CCT3), NM_006430 (CCT4), NM_012073 (CCT5), NM_001762 (CCT6), NM_006429 (CCT7), and NM_006585 (CCT8). The cDNA for each subunit was inserted into a pM vector (Clontech), respectively, encoding the GAL4 DNA binding domain. The full-length and four types of truncated cDNAs of AIB1 (GenBank accession no. NM_006534) were amplified from MCF-7 cells by RT-PCR, subcloned in-frame into the pVP16 vector (Clontech) encoding the VP16 transactivation domain, and verified by sequencing. pG5CAT reporter vectors (0.5 µg), containing a chloramphenicol acetyltransferase (CAT) reporter gene under the control of the GAL4 response element and 2.5 µg of each of the above-mentioned constructed vectors, were co-transfected into 2.5×10^5^ MCF-7 cells per well in 6-well plates using the LF2000 reagent (GIBCO BRL). After 48 h, the cells were harvested and the extracts were assayed for CAT activity using CAT ELISA assay kits (Roche).

### Stable Transfection and Selection of CCTζ-, AIB1-, and ERα-transfected Cells

The pIRES expression vector contained a cytomegalovirus promoter and pIRES-CCTζ, pIRES-AIB1, and pIRES-ERα, encoding the human CCTζ, AIB1, and ERα proteins, respectively. The full-length cDNA of CCTζ, AIB1, or ERα was amplified by PCR, inserted into the pIRES plasmids with *Cla*I and *Xba*I sites, and were confirmed by DNA sequencing. Transfection was carried out using Lipofectin (Life Technologies) in accordance with the manufacturer instructions. MCF-7 cells cultured in 6-cm dishes were washed twice and supplemented with 3 mL Opti-MEM-reduced serum medium. The pIRES-CCTζ, pIRES-AIB1, pIRES-ERα, or pIRES plasmid DNA (2 µg per 6-cm dish) was mixed with Lipofectin before addition to MCF-7 cells. After transfection, stable transfectants were selected by incubating with 500 µg/mL geneticin (G418; Sigma-Aldrich). The surviving colonies were picked out ∼2 weeks later, and the CCTζ, AIB1, and ERα expression levels were determined by Western blotting. Positive clones were maintained in culture medium supplemented with 250 µg/mL G418.

### Preparation of shnRNA Vectors, Transfection, and Stable Cell Lines

RNA interference (RNAi) was performed as described previously [16] using the pSilencer 3.1H1 hygro vector (Ambion; Austin, TX, USA) to direct the relevant hairpin double-stranded RNAs. The sequence of small interfering RNA (siRNA) target sites for CCTζ, AIB1, and ERα were designed by siRNA Design (Ambion). A sequence of 19 nucleotides (CCUCA CUUGU AACGU GUCA in CCTζ, GCGAA GUUUA AUGAU CCAC in AIB1, and GUGGA UCAUU AAACU UCGC in ERα) were determined and compared with the nucleotide database using BLAST (www.ncbi.nlm.nih.gov/BLAST). The hairpin siRNA template oligonucleotides were chemically synthesized by Invitrogen (Shanghai, China), annealed, and cloned into the pSilencer 3.1H1 hygro vector between the *Bam*HI and *Hind*III digestion sites, designated as siCCTζ (pSilence-CCTζ), siAIB1 (pSilence-AIB1), and siERα (pSilence-ERα). The control pNegative vector (negative control of the pSilencer 3.1H1 hygro vector with limited homology to any known sequences in the human genome) was provided by Ambion. The positive constructs were validated by sequencing. Each construct (2.5 µg) was transfected into 2.5×10^5^ MCF-7 and T47D cells per well with FuGene6 reagent (Roche; Branchburg, NJ, USA) according to manufacturer instructions. MCF-7 and T47D cells were transfected with the pSilence-CCTζ or pSilence-AIB1 expression plasmids. Stable transfections were obtained by sustained selection with 200 µg/mL hygromycin B (Stratagene; La Jolla, CA, USA). Positive clones of MCF-siCCTζ, MCF-siAIB1, T47D-siCCTζ, T47D-siAIB1, or the pNegative vector (clones MCF-siV and T47D-siV) were maintained in culture medium supplemented with 200 µg/mL hygromycin B (Stratagene).

### Real-time RT-PCR

Total RNA was extracted and DNase was treated with the RNeasy Mini kit (Qiagen). Real-time RT-PCR was conducted with the SuperScript One-Step Reverse Transcription-PCR with Platinum Taq system (Invitrogen). Samples were reverse transcribed for 30 min at 58°C, followed by a denaturing step at 95°C for 5 min and 40 cycles of 15 s at 95°C and 1 min at 58°C. Fluorescence data were collected during the 58°C step with the Cycler iQ Detection System (Bio-Rad Laboratories; Hercules, CA). The primers and probes for real-time RT-PCR measurements were as follows: c-myc forward primer, 5′-CCAGG ACTGT ATGTG GAGCG-3′ and reverse primer, 5′-CCTGAGGACCAGTGGGCTGT-3′; cyclin D1 forward primer, 5′-CTGGC CATGA ACTAC CTGGA-3′ and reverse primer, 5′-GTCAC ACTTG ATCAC TCTCC-3′; PgR forward primer, 5′-GCATC AGGCT GTCAT TATGG-3′ and reverse primer, 5′-AGTAG TTGTG CTGCC CTTCC-3′.

### Ubiquitination Assays

*In vivo* ubiquitination assays, after immunoprecipitation by AIB1 antibody or IgG, ubiquitinated AIB1 was detected by ubiquitin antibodies in Western Blot.

### Statistical Analyses

Data are presented as mean ± S.E.M. from at least three to eight independent experiments. Student’s unpaired *t*-tests (two-tailed) were used to determine statistical differences in promoter activities. Differences were considered statistically significant at P<0.05.

## Results

### Substrate Rigidity Affects MCF-7 Spreading, Proliferation, and Cell Cycle

To address how the biological behavior of breast cancer cells could be governed by substrate rigidity, ERα-positive breast cancer cells (MCF-7) were plated on 10-, 30-, and 100-kPa substrates. The morphology of the breast cancer cells clearly differed on the silicone substrates of different rigidity. The density of cells growing on the 100-kPa substrate was much higher than that on the 10-kPa and 30-kPa silicone substrates after culturing for 120 h (Fig. 2). The cell spreading area on the 100-kPa silicone substrate was also greater than that of cells incubated on the 10- and 30-kPa substrates after 24 to 144 h culture (Fig. 3A). We also observed that the growth rate of MCF-7 cells was higher on 100-kPa substrates than on 10-kPa and 30-kPa substrates (*P*<0.01, Fig. 3B). In addition, the percentage of cells in the DNA synthesis phase of the cell cycle was higher in the MCF-7 cell line growing on the hard rigidity substrate (100 kPa) compared to those grown on the softer substrates (10 kPa and 30 kPa), which was predominantly due to a reduction of the G0/G1 phase and increased G2/M phases of the cell cycle (*P*<0.01, Fig. 3C, D, E and F). Altogether, these results indicate that breast cancer cells were able to sense and respond to the rigidity of their substrates, and that substrate rigidity could affect cell spreading and proliferation.

**Figure 2:** Growth characteristics and morphology of cells grown on different rigidity silicone substrates, E_Y_ = 10, 30 and 100 kPa (×400). E_Y_: the Young’s modulus.

**Figure 3:** Effects of substrate rigidity on cell proliferation, spreading area, and cell cycle in the MCF-7 breast cancer cells. (**A**) The cellular spreading area of MCF-7 cells grown on different rigidity substrates for different lengths of times. Data are presented as the means ± SEM from three independent experiments. **P<0.01. (**B**) The proliferation rate of MCF-7 cells grown on different rigidity substrates for different lengths of time. Data are presented as the means ± SEM from three independent experiments. **P<0.01. (**C–E**) Cell cycle analysis of MCF-7 cells grown on different rigidity substrates in three independent experiments. **P<0.01. (**F**) MCF-7 cells grown on different rigidity substrates for 120 hours; data show the results of flow cytometry plots from one of three independent experiments.

### Chaperonin CCT Expression in MCF-7 Cells Increased on Harder Substrates

To obtain a global perspective of the molecular pathways involved in the response to substrate rigidity, we employed SILAC in conjunction with LC-MS/MS to assess the rigidity-induced differential expression of the whole proteome of MCF-7 cells for 72 h, and the lysates were combined and subsequently fractionated by SDS-PAGE. After in-gel digestion, the proteins were identified and quantified by LC-MS/MS. The experimental scheme is shown in Fig. 1. By using SILAC and a database search, more than 2125 and 2312 proteins were quantified. Of these identified proteins, 1735 proteins appeared in both extracts, and 151 of these proteins were differentially regulated by the different rigidity substrates (10 and 100 kPa), Fig. S1. The proteins were filtered by their significance thresholds (P<0.05), and the peptide spectra were compared to quality threshold values. Following these quality control steps, data revealed that all eight subunits of chaperonin CCT were significantly increased by 1.94- to 2.198-fold on the hardest substrate (100 kPa) compared to the softest substrate (10 kPa) (Table 1). To explore this interesting phenomenon further, we here focus on the functions of chaperonin CCT in rigidity-induced breast cancer cell proliferation. The global data describing the proteome expression of cells grown on different rigidity substrates will be published in a separate manuscript.

**Table 1:** SILAC results showing that eight CCTs members were closely related to the cell’s rigidity response to 10-kPa (Protein Label Light media) and 100-kPa (Protein Label Heavy media) substrates.

Protein IDs	Protein Names	Gene Names	Proteins	Peptides	Unique Peptides	Ratio H/L Normalized	Ratio H/L Variability [%]	Ratio H/L Count
IPI00027626	CCT-zeta-1;TCP 1 subunit zeta	CCT6;CCT6A;CCTZ	5	13	13	2.1308	8.3862	13
IPI00784090	CCT-theta; TCP 1 subunit theta	CCT8;CCTQ	4	16	16	2.1983	13.52	9
IPI00553185	CCT-gamma;TCP 1 subunit gamma	CCT3;CCTG	6	9	9	2.1225	4.1895	5
IPI00018465	CCT-eta;TCP 1 subunit eta	CCT7;CCTH	5	16	16	2.0743	11.219	15
IPI00010720	CCT-epsilon;TCP 1 subunit epsilon	CCT5;CCTE	3	10	9	2.0742	83.56	12
IPI00302927	CCT-delta;TCP 1 subunit delta	CCT4;CCTD	3	13	12	1.94073	10.918	5
IPI00297779	CCT-beta;TCP 1 subunit beta	CCT2;CCTB	2	20	20	1.99446	10.537	19
IPI00290566	CCT-alpha;TCP 1 subunit alpha	CCT1;CCTA;TCP1	2	11	11	2.0765	7.7885	8

TCP1:T-complex protein 1.

We used Western Blot and Real-time RT-PCR to detect chaperonin CCT mRNA and Protein expression levels in breast cancer cells grown on substrates of different rigidity (10, 30, and 100 kPa). The results showed that in both MCF-7 and T47D cells, the expressions of chaperonin CCTα, CCTβ, CCTγ, CCTδ, CCTε, CCTζ, CCTη, and CCTθ were higher on harder substrates than on softer substrates (Fig. 4A, B and C). Then, we detected the chaperonin CCT folding activity of denatured β-actin in MCF-7 cell extracts growing on different substrates (10 kPa, 30 kPa, 100 kPa) to determine whether the expression levels of chaperonin CCTs on hard substrates was proportional to the folding activity. The results showed that chaperonin CCTs’ folding activity was also significantly increased on the harder substrate (100 kPa) compared to the softer substrates (10 kPa and 30 kPa) (Fig. 4D). However, whether chaperonin CCT plays a role in hard substrate-induced MCF-7 proliferation is yet to be elucidated.

**Figure 4:** Effects of substrate rigidity on the mRNA and protein expression levels of CCTs, and changes in CCT folding activity. (**A**) Western Blot analysis showing changes in the protein expression of CTT/TRiC in the breast cancer cell line MCF-7 cultured on 10-kPa, 30-kPa, and 100-kPa substrates, respectively. (**B**) Western Blot showing changes in the protein expression of CT/TRiC in the breast cancer cells T47D cultured on 10, 30, and 100-kPa substrates. (**C**) Real-time RT-PCR showing changes in the mRNA expression of CTTs in MCF-7 and T47D breast cancer cells cultured on 10, 30, and 100 kPa substrates, **P<0.01, compared with 10 or 30 kPa substrates. (**D**) CCTs folding activity in MCF-7 cell extracts grown on different substrates (10, 30, and 100 kPa).

### CCTζ Subunit Binding and the Folding of AIB1 occurs via PFD- and ERα-independent Pathways

Previous studies demonstrated that chaperonin CCT mostly recognize proteins containing large β-pleated sheet structures, such as actin, tubulin, G protein β subunit (Gb), and VHL [17], [18], and that CCTζ also recognizes some polyglutamine-expanded proteins [19]. CCT is involved in the oncoprotein cyclin E, the Von Hippel-Lindau tumour suppressor protein, cyclin B and p21^(ras)^ folding which strongly suggests that it is involved in cell proliferation and tumor genesis [20], [21]. To test our hypothesis that chaperonin CCTs play a role in promoting the growth of ERα-positive breast cancer cells on harder substrates, we used bioinformatic analyses to screen ERα and ERα-related co-activators that contain polyglutamine-repeat domains, and identified AIB1 [22].

As shown in Fig. 5A, only AIB1, and not ERα, was identified in the protein complex by using anti-CCTη or anti-CCTζ antibodies for immunoprecipitation, suggesting that chaperonin CCT could potentially interact with AIB1 in breast cancer cells. Furthermore, the mRNA and protein expressions of AIB1 in both MCF-7 and T47D cells were higher on the harder substrate (100 kPa) compared to the softer substrates (10 kPa and 30 kPa) (Fig. 5B and C). In addition, AIB1 folding activity was induced to a greater extent in MCF-7 cells growing on the harder substrate (100 kPa) than on the softer substrates (10 kPa and 30 kPa), as shown in Fig. 5D. Conversely, the depletion of CCTζ inhibited AIB1 folding activity, which suggested that the AIB1 folding activity was CCTζ-dependent (Fig. 5E).

**Figure 5:** CCT6 (ζ) interacts with AIB1, and stimulates AIB1 refolding via a PFD-independent pathway. (**A**) MCF-7 cells were cultured on 100-kPa substrates, and then analyzed by co-immunoprecipitation (co-IP) assay followed by immunoblotting (IB) analysis after 72 h. (**B**) The expression of AIB1 was then assessed in two breast cancer cell lines (MCF-7 and T47D) grown on different rigidity substrates using Western Blotting. GAPDH was used as a control to confirm equal protein loading. Each lane was loaded with up to 30 µg of protein. (**C**) The mRNA expression of *AIB1* in MCF-7 and T47D breast cancer cells grown on different rigidity substrates was assessed using real-time RT-PCR. **P<0.01 compared with 10 and 30 kPa substrates. (**D**) Altered CCTs folding activity on AIB1 changes in the MCF-7 cells grown on different rigidity substrates (10 kPa, 30 kPa, 100 kPa). (**E**) MCF-7 cell extracts were assayed before and after CCTζ, ERα, and PFD immunodepletion assayed using [^35^S]-labeled, and denatured AIB1 (500 ng per lane). The protein concentration of MCF-7 cells was 2.5 mg/mL. PFD immunodepletion did not affect AIB1 refolding. therefore, CCTs folded AIB1 in a PFD-independent pathway. (**F**) The levels of CCTζ, ERα, and PFD were measured in MCF-7 cell extracts after immunodepletion. (**G**) Ubiquitinated forms of AIB1 in cells grown on different rigidity substrates with ERα or CCTζ overexpression or knockdown were detected using co-immunoprecipitation (co-IP) with anti-AIB1 antibodies and Western blotting with anti-ubiquitin antibodies.

There are two pathways for chaperonin CCT-mediated protein folding: PFD-dependent or independent. Therefore, we assessed the pathway used for chaperonin CCT-mediated AIB1 folding activity by depleting PFD (Fig. 5E), and the results suggested that chaperonin CCT-mediated AIB1 folding activity occurs via a PFD-independent pathway.

PFD is a dedicated CCT co-chaperone for folding proteins. Eukaryotic PFD forms jellyfish-shaped hexameric complexes consisting of two α-type and four β-type subunits, with six unique subunits in eukaryotes. The six tentacle-like PFD subunits form a rectangular cavity, which binds the partially folded chains of proteins emerging from the ribosome before delivering them to CCTs. Yeast cells lacking PFD function fold actin and tubulin more slowly compared to wild-type cells.

In this study, immuno-depletion of ERα and PFD had no effect on AIB1 folding. By contrast, CCTζ immuno-depletion from a cell extract where it was significantly expressed, such as MCF-7, led to a dramatic decrease in AIB1 folding. This strongly suggests that CCTζ plays a role in modulating AIB1 folding.

### CCTζ Binds to the Polyglutamine Repeat Domain of AIB1

We next used mammalian two-hybrid protein-protein interaction assays to identify the subunit of chaperonin CCT that binds with AIB1 to further investigate the interaction *in vivo* and to delineate the binding activities. We constructed all eight full-length chaperonin CCT subunits (α to θ) and AIB1, and found that AIB1, both alone and when co-transfected with CCTα, β, γ, δ, ε, η, or θ into MCF-7 cells, could not stimulate the expression of the CAT reporter gene. The expression of the CAT reporter gene was only significantly stimulated when AIB1 and CCTζ were co-transfected into MCF-7 cells (Fig. 6A).

**Figure 6:** Binding activities of CCTs and AIB1 in MCF-7 cells. (**A**) The reporter plasmid pG5CAT, expressing CAT, was co-transfected with the pM construct of CCT (α, β, γ, δ, ε, ζ, η or θ) and the pVP16 construct of AIB1 into MCF-7 cells. In the presence of pG5CAT, the control cells were only transfected with the pVP16 construct of AIB1, respectively. CAT activities were measured at a wavelength of 415 nm. Error bars show the standard deviations (n = 6, **P<0.01, compared with other columns). (**B**) The molecular structure of AIB1, and the constructed fusion proteins in the mammalian two-hybrid protein-protein interaction system were used to compare the binding activities between CCT and AIB1 or truncated forms of AIB1. The numbers at the top indicate the position of the amino acid sequence. The letters within the bar indicate structural domains, and the lines under the bar indicate functional domains. bHLH, basic helix-loop-helix domain; L, LXXLL α-helix motif; S/T, serine/threonine-rich region; Q, glutamine-rich domain. (**C**) Binding activities of CCTζ and AIB1 or four truncated forms of ΔAIB1 (a to d) in MCF-7 cells. The constructed fusion proteins in the mammalian two-hybrid protein-protein interaction system were used to compare the binding activities between the full-length CCTζ and wild-type AIB1, or truncated forms of AIB1. The reporter plasmid pG5CAT was co-transfected with the pM construct of CCTζ and the pVP16 construct of AIB1 or the four types of truncated AIB1 into MCF-7 cells. In the presence of pG5CAT, two control cell lines were only transfected with the pVP16 construct of AIB1 or the pM construct of CCTζ, respectively. Error bars show standard deviations (n = 3) of three independent experiments in duplicate (**P<0.01, column 3, 4 or 7 vs. column 5 or 6).

To identify the binding domain for AIB1 binding to CCTζ, we constructed a full-length AIB1 vector and four vectors expressing truncated forms of AIB1 (ΔAIB1*a* 1272–1420 amino acids (aa); ΔAIB1*b* 1244–1420 aa; ΔAIB1*c* 580–1420 aa; ΔAIB1*d* 1–950 aa; Fig. 6B). The results showed that the full-length AIB1, ΔAIB1*a*, and ΔAIB1*d*, containing the polyglutamine repeat domain, could bind to CCTζ and stimulated the expression of the CAT gene, increasing the activity by at least 3-fold compared with ΔAIB1*b* or ΔAIB1*c* binding to CCTζ (Fig. 6C). These results suggest that the polyglutamine repeat domain (contained in AIB1, ΔAIB1*a*, and ΔAIB1*d*) is an important factor that regulates the expression of the CAT reporter gene, and that the polyglutamine repeat domain of AIB1 is essential for the physical interaction between CCTζ and AIB1.

### CCTζ-mediated AIB1 Folding is Involved in the Cellular Rigidity Response of MCF-7 Cells

To investigate the role of CCTs and AIB1 in the rigidity response of MCF-7 cells, we established several MCF-7 cell clones: stable AIB1-overexpressing MCF-7 cells (clone ovAIB1), stable AIB1-silenced MCF-7 cells (clone siAIB1) (Fig. 7A and B), stable CCTζ-overexpressing MCF-7 cells (clone ovCCTζ), stable CCTζ-silenced MCF-7 cells (clone siCCTζ) (Fig. 7A and C), AIB1-overexpressing and CCTζ-silenced MCF-7 cells (clone ovAIB1+siCCTζ), and CCTζ-overexpressing and AIB1-silenced MCF-7 cells (clone ovCCTζ+siAIB1) (Fig. 7A and D). All cells were seeded on the 100-kPa substrate and cell growth characteristics were assessed. The results showed an increase in the cell area in the AIB1-overexpressing group compared with the other groups, particularly the ovAIB1+siCCTζ group. This suggests that AIB1 plays an important role in increasing the cell area, and that this role is CCTζ-dependent. The results also showed that in the siAIB1, siCCTζ, ovAIB1+siCCTζ, and ovCCTζ+siAIB1 groups, the cell area was reduced compared with the control, which indicates that the increase in cell area induced by the hard substrate was related to CCTζ-AIB1.

**Figure 7:** Effects of the overexpression and/or knock-down of AIB1 and/or CCTζ on the cell proliferation, spreading area, and cell cycle of breast cancer MCF-7 cells grown on silicone substrates with E_Y_ = 100 kPa (**P<0.01). (**A**) The mRNA expression levels of AIB1 and CCTζ in control, siAIB1, ovAIB1, siCCTζ, ovCCTζ, siAIB1+ovCCTζ, and siCCTζ+ovAIB1 MCF-7 cell groups were validated by real-time RT-PCR, **P<0.01, compared with control cells. (**B**) The expression of AIB1 in the siAIB1 and ovAIB1 MCF-7 cell was validated by Western Blot. (**C**) The expression of CCTζ in the siCCTζ and ovCCTζ MCF-7 cells was validated by Western Blot. (**D**) The expression of AIB1 and CCTζ in the siAIB1+ovCCTζ and siCCTζ+ovAIB1 MCF-7 cells was validated by Western Blot. (**E**) The spreading area of all Cell types (control, si-AIB1, si-CCTζ, ovAIB1, ovCCTζ, si-AIB1+ovCCTζ, and siCCTζ+ovAIB1) grown on silicone substrates with E_Y_ = 100 kPa. **P<0.01. (**F**) Growth curves of all cells (control, siAIB1, siCCTζ, ovAIB1, ovCCTζ, siAIB1+ovCCTζ, and siCCTζ+ovAIB1) grown on silicone substrates with E_Y_ = 100 kPa. **P<0.01. G2/M phase (**G**), G0/G1 phase (**H**), and S phase (**I**) of the cell cycle was assessed in cells (control, si-AIB1, siCCTζ, ovAIB1, ovCCTζ, siAIB1+ovCCTζ, and siCCTζ+ovAIB1) grown on silicone substrates with E_Y_ = 100 kPa. **P<0.01 compared with si-AIB1.

The growth curve analysis demonstrated that proliferation increased significantly in the ovAIB1 group compared with the other groups. The growth rate decreased in the siAIB1, siCCTζ, ovAIB1+siCCTζ, and ovCCTζ+siAIB1 groups of MCF-7 cells, which tended to correspond with cell area changes. These results suggest that the higher expression levels of chaperonin CCT and the increased ability of AIB1 folding are related to the MCF-7 response to hard substrates (Fig. 7E, F, G, H and I).

The percentage of cells in the DNA synthesis phase of the cell cycle was higher in the ovAIB1 group compared to those in the siAIB1, siCCTζ, ovAIB1+siCCTζ, and ovCCTζ+siAIB1 groups of MCF-7 cells. Accordingly, the percentage of cells in the G0/G1 phase was lower in the ovAIB1 group than in the other groups, and that in G2/M phases was higher than others. (*P*<0.01, Fig. 7G–I).

### AIB1 and ERα Co-regulated Genes Involved in the Proliferation of MCF-7 Cells

We next assessed the mRNA and protein expression of c-Myc, cyclin D1, and PgR, which are all co-regulated by ERα and AIB1, to further investigate the mechanism underlying the role of CCT-mediated AIB1 folding in the rigidity-induced proliferation of MCF-7 cells [23]. The results demonstrated that the expressions of the *c-myc*, *cyclin D1*, and *PgR* genes was higher on hard substrates than on soft substrates in both MCF-7 and T47D cells (Fig. 8A and B). ERα and AIB1 could up-regulate both the mRNA and protein expressions of the c-myc, cyclin D1, and PgR genes, and these effects were enhanced by 17 β-estradiol (E2). In addition, the anti-estrogen, 4-hydroxytamoxifen (4HT), could significantly inhibit the ERα and AIB1-stimulated up-regulation of the mRNA and protein expressions of the c-myc, cyclin D1, and PgR (Fig. 8C and D).

**Figure 8:** The mRNA and protein expression of the c-myc, cyclin D1, and PgR, which are co-regulated by ERα and AIB1. Western blotting for the protein expression of cyclin D1, c-myc, and PgR in MCF-7 (**A**) and T47D (**B**) cells grown on different rigidity silicone substrates for 48 h. (**C**) Real-time RT-PCR analysis of the mRNA expression of the *c-cmy*, *cyclin D1*, and *PgR* genes in siAIB1, siERα, ovAIB1, ovERα, siAIB1+ovERα, siERα+ovAIB1, and control MCF-7 cells grown on 100-kPa silicone substrate for 48 h. Data were calculated relative to GAPDH expression and are presented as mean ± SD fold-change compared with wild MCF-7 control cells (n = 3); **P<0.01, compared with control cells; ^##^P<0.01, compared with the siAIB1, siERα, siAIB1+ovERα, and siERα+ovAIB1 MCF-7 cells. (**D**) The siAIB1, siERα, ovAIB1, ovERα, siAIB1+ovERα, siERα+ovAIB1, and wild MCF-7 cells grown on the 100-kPa silicone substrate for 48 h. Crude proteins were then extracted from the cells were subjected to SDS-PAGE followed by Western immunoblot with the antibodies against c-myc, cyclin D1, and PgR. (**E**) The protein expression of ERα and AIB1 in siAIB1, siERα, ovAIB1, ovERα, siAIB1+ovERα, siERα+ovAIB1, and wild MCF-7 cells by Western blot.

## Discussion

The most common metastasis site of breast cancer is the bone [24], and majority of breast cancers that metastasize to the bone are ERα-positive cells [25]. Current treatments with bisphosphonates have greatly reduced the number of skeletal-related events experienced by breast cancer patients; however, because there are no effective treatments to inhibit tumor growth, bone metastases remain incurable [26http://www-ncbi-nlm-nih-gov.ezproxyhost.library.tmc.edu/pmc/articles/PMC3234324/- CR1]. Therefore, there is clinical importance to investigate the mechanisms of bone metastasis in breast cancer.

It is currently well accepted that tumor cells are influenced by other cells and growth factors present in the bone microenvironment, which lead to tumor-induced bone disease. Many research groups have studied this process and determined the major contributing factors; however, the results obtained thus far cannot fully explain the changes in gene expression and cell behavior that occur when tumor cells metastasize to the bone [27]. More recently, many studies have shown that mechanical properties of the matrix environment play a significant role in regulating the proliferation and morphological properties of cancer cells [28]. Cellular responses to the mechanical rigidity of the extracellular matrix are correlated with the rigidity of the target tissue and the rigidity of the microenvironment, which might regulate tumor cell behavior and gene expression [29]. Therefore, we hypothesized that the cellular response to rigidity was related to the high incidence of bone metastasis in breast cancer.

In this study, we used ERα-positive human breast cancer cells (MCF-7) in a variety of assays where the substrate rigidity was varied to mimic the environment that these cells might encounter *in vivo*. We found that the rigidity of the substrate affected cell growth, and that ERα-positive human breast cancer cells exhibited increased proliferation and spreading ability on harder substrates (Fig. 2 and 3). Therefore, at least some ERα-positive human breast cancer cells are more likely to grow on highly rigid substrates. Bone is a unique microenvironment compared with all other tissues in the body, and is more rigid than normal breast tissue [27]. Our results demonstrated that the growth rate of ER-negative cells (MD-MDA-435 and BT549) did not significantly change on different rigidity of matrix (Fig. S2A and B). Therefore, we hypothesized that the high incidence of bone metastasis in ERα-positive breast cancer could be explained by the preferential growth of ERα-positive human breast cancer cells on rigid substrates.

To further investigate why ERα-positive human breast cancer cells preferentially grow on hard substrates, we used SILAC to compare the whole proteome of breast cancer cells grown on different rigidity substrates. The cytosolic chaperonin complex, chaperonin containing t-complex protein 1 (CCT), chaperonin containing T-complex polypeptide 1 (TCP-1), or the so-called TCP-1 ring complex (TRiC) was identified. Eight CCT members (CCTα to θ) were found to show two times higher expression on hard substrates (Table 1). The chaperonin CCT is a highly conserved molecular chaperone, and the main function of CCT is to promote the correct folding of newly synthesized proteins or the refolding of some misfolded proteins [30]. CCT is a 16-subunit complex composed of two back-to-back stacked rings, each containing eight different subunits of approximately 60 kDa (α, β, γ, δ, ε, ζ, θ, and η). Each CCT subunit contains a different substrate-binding site, which specifically binds to different proteins prior to regulating their folding. Unlike most molecular chaperones, CCT is not induced by stress, but is instead transcriptionally and functionally linked to protein synthesis [31]. The molecular chaperone CCT plays a central role in maintaining cellular proteostasis and is involved in folding oncoprotein cyclin E, the Von Hippel-Lindau tumor suppressor protein, cyclin B, and p21^ras^, which suggests that it might play a role in cell proliferation and tumorigenesis. In the present study, CCT expression was higher on the 100-kPa substrate than on the 10-kPa and 30-kPa substrates in both MCF-7 and T47D cells (Fig. 4 A, B and C). In addition, the CCT folding activity was found to increase on hard substrates compared with softer substrates (Fig. 4D). Our results suggest that the high rigidity of substrates could induce CCT expression and enhance its folding activity. Therefore, CCT might play some role in the preferential growth of ER-positive breast cancer cells on hard substrates.

Previous studies have demonstrated that CCT chaperonins play an essential role in the modulation of folding polyglutamine-expanded proteins [15]. CCTs might specifically recognize not only the β-strand of the polyglutamine tract but also the context structure surrounding the polyglutamine tract of each different protein. To identify the functional protein downstream of CCT in hard substrate-induced cell proliferation, we used the bioinformatics method to screen for proteins containing polyglutamine repeat sequences (CCT binding domain) with a function related to ERα. AIB1 was found to meet the above conditions, containing a polyglutamine domain and being a member of the p160 steroid receptor co-activator family, which mediates the transcriptional activities of nuclear receptors including the ER and progesterone receptor (PR) [32]. The results of this study demonstrated that chaperonin CCT could potentially interact with AIB1 (Fig. 5A). In addition, high substrate rigidity could enhance AIB1 protein and mRNA expressions (Fig. 5B and C) and increase CCTζ folding activity for AIB1 (Fig. 5D), and the folding activity occurred via a PFD- and ERα-independent pathway (Fig. 5E and F). In addition, AIB1 ubiquitination did not change significantly in cells grown on different rigidity substrates. There was also no obvious change in AIB1 ubiquitination in cells in which ERα and CCTζ were overexpressed or knocked down (Fig. 5G).

Actin and tubulin appear to have co-evolved with at least two molecular chaperones that are specifically required for their biogenesis: (PFD) and chaperonin CCT [33]. Previous studies demonstrated that PFD binds to nascent polypeptides at the ribosome, and maintains them in a folding-competent state until they can deliver to CCT for folding in a protected compartment [34], [35]. PFD overexpression has been observed in many tumor types, including pancreatic cancer and neuroblastoma [36], [37], whereas CCT overexpression has been observed in liver cancer and in the late stages of colon cancer [38], [39]. Taken together, these findings suggest that PFD and CCT play roles in uncontrolled cell proliferation, and that the link between CCT/PFD and cancer might be related to tubulin biogenesis. Nevertheless, there is no conclusive evidence that proteins (such as VHL, c-Myc, and MSH4) other than actin and tubulin can bind to individual subunits of PFD [40], [41], [42]. Therefore, we designed this study to assess the role of PFD in CCT-mediated folding of the previously unidentified substrate AIB1.

Then, we screened the interactions of eight chaperonin CCT subunits (α, β, γ, δ, ε, ζ, η, or θ) with AIB1 by using the mammalian two-hybrid protein-protein interaction system, and found that only the CCTζ subunit could bind to AIB1 (Fig. 6A), whereas none of the other subunits could. We designed four truncated forms of AIB1 (Fig. 6B) and measured their binding to CCTζ, and found that the polyglutamine repeat sequence of AIB1 is essential for the physical interaction between AIB1 and CCTζ (Fig. 6C). Furthermore, CCTζ-mediated AIB1 folding was shown to be heavily involved in the response to cellular rigidity response (*P*<0.01, Fig. 7). Overexpression of AIB1 and CCTζ have same effects on soft substrates with E_Y_ = 10 kPa as on hard substrates with E_Y_ = 100 kPa (Fig. 7 and Fig. S4). This strongly suggests that the CCT-AIB1 interaction plays a role in ERα-positive breast cancer cells that preferentially grow on hard substrates. We also assessed the relationship between AIB1 with ERα, and results showed that the overexpression of AIB1 or ERα in MCF-7 cells promoted cell proliferation; conversely, when the expression of AIB1 or ERα was knocked down, the overexpression of ERα or AIB1 had no effect on cell proliferation (Fig. S2 C and D).

The biological contribution of 17β-estradiol (E2) to the initiation and progression of breast cancer is widely accepted [43]. Estrogens act by binding to nuclear ERs, ERα or ERβ, which function as ligand-regulated transcription factors. Liganded ERs dimerize and bind to estrogen response elements (EREs). The ER complex is then able to recruit co-activators that are involved in enhancing ER-mediated gene transcription and the expression of target genes [44]. The best-characterized co-activator proteins associated with ER signaling belong to the p160 steroid receptor co-activator (SRC) family comprising three members, SRC-1, SRC-2, and SRC-3. AIB1 (also known as SRC-3) was identified as a gene that is frequently amplified in breast cancer [45]. AIB1 plays a central role in promoting cell proliferation, migration, invasion, and metastasis by signaling through ERα, as well as by activating the growth factor receptors human epidermal growth factor receptor 2 (HER2), epidermal growth factor receptor (EGFR), and insulin-like growth factor receptor (IGFR) [46]. In addition, AIB1 depletion blocked estradiol-stimulated cell proliferation [47]. The results of *in vivo* studies demonstrated that a knockout of AIB1 suppressed mammary tumor initiation, growth, and metastasis [48], whereas forced expression in mouse mammary epithelial cells was sufficient to induce spontaneous mammary tumorigenesis [49]. We assessed the binding activities of CCTs with SRC1 and SRC2 in MCF-7 cells, and the results demonstrated that CCTs had a lower binding affinity for SRC1 or SRC2 than AIB1 (Fig. S3). The differences in the length and sequences of the Q-rich domain (glutamine-rich region) among SRC1, SRC2, and AIB1 are shown below (Q, glutamine):

SRC1: NIGGQFGTGINPQMQQNVFQYPGAGMVPQGEANFAPSL (1212–1249 aa glutamine-rich region sequences) http://www.ncbi.nlm.nih.gov/protein/AAI11534.1.

SRC2:MPATMSNPRIPQANAQQFPFPPNYGISQQPDPGFTGATTPQSPLMSPRMHTQSPMM (1281–1338 aa glutamine-rich region sequences) http://www.ncbi.nlm.nih.gov/protein/NP_006531.1.

SRC3:MDGLLAGPTMPQAPPQQFPYQPNYGMGQQPDPAFGRVSSPPNAMMSSRMGPSQNP (1289–1344 aa glutamine-rich region sequences) http://www.ncbi.nlm.nih.gov/protein/AAH92516.1.

These differences in the length and sequences of SRC1, SRC2, and AIB1 might partly explain the different binding activities between CCTs and SRCs. In addition, SRC1, SRC2, and AIB1 exhibit different biological functions. For example, Carroll et al reported that genes that are bound by SRC3 and ERα, but not other p160 proteins, have predictive value in a cohort of breast cancer patients [50].

In estrogen-responsive breast cancer cells, E2 induces cell proliferation by stimulating progression through the G1 phase of the cell cycle [51.]. Many of the genes involved in cell growth, growth factor signaling, and cell cycle control are estrogen-responsive (e.g., the cyclin D1, c-myc, and PgR genes) [52]. For instance, an increase in cyclin D1 levels is found in 10–15% of invasive breast carcinomas and appears to be an early event in the development of breast carcinoma [53], [54]. Furthermore, Tamoxifen, an ERα antagonist, which inhibits ERα-dependent gene expression and consequently cell growth, is used therapeutically for breast cancer [55].

Our data in both MCF-7 and T47D cells suggest that the mRNA expressions of the *c-myc*, *cyclin D1*, and *PgR* genes were higher on hard substrates than on soft substrates (Fig. 8A and B). The mRNA and protein expressions of the c-myc, cyclin D1, and PgR genes are co-regulated by ERα and AIB1 (Fig. 8C and D); therefore, the E2-ERα/AIB1-c-myc, cyclin D1, and PgR pathways are likely to be involved in the preferential growth of ERα-positive breast cancer cells on hard substrates. Moreover, these effects were significantly enhanced in the presence of E2, whereas the ERα antagonist, 4HT, weakened these effects significantly (Fig. 8C and D). Nevertheless, we were unable to explain why the overexpression of ER combined with siAIB1 inhibited the functionality of ER, since siAIB1 without the overexpression of ER had no effect (Fig. 8D). These observations will be explored further in future studies.

## Conclusion

In summary, this study demonstrates that ERα-positive breast cancer cells grow preferentially on hard substrates. Chaperonin CCT-mediated AIB1 folding is involved in the rigidity response of breast cancer cells and regulates the ERα/AIB1-c-myc, cyclin D1, and PgR pathway. These important observations provide novel insight into the mechanisms of bone metastasis.

## Supporting Information

Figure S1 **The log_2_ fold change of 151 differentially expressed proteins.**
(TIF)

Figure S2 **Effects of substrate rigidity on the proliferation of MDA-MB-435 and BT549 breast cancer cells (ERα negative cells).** (**A**) The proliferation rate of MDA-MB-435 cells grown on different rigidity substrates for varying lengths of time. Data are presented as the means ± SEM of three independent experiments. (**B**) The proliferation rate of BT549 cells grown on different rigidity substrates for varying lengths of time. Data are presented as the means ± SEM of three independent experiments. (**C**) Effects of the overexpression and/or knock down of AIB1 and/or ERα on the proliferation of MCF-7 breast cancer cells grown on silicone substrates with E_Y_ = 100 kPa, and with 10 nM E2. **P<0.01, ovAIB1 and ovERα compared with siAIB1, siERα, siAIB1+ovERα, and siERα+ovAIB1; ^#^ *P*<0.05, compared with control. (**D**) Effects of the overexpression or knock down of AIB1 and/or ERα on the proliferation of MCF-7 breast cancer cells grown on silicone substrates with E_Y_ = 100 kPa in the presence of 4HT.
(TIF)

Figure S3 **The binding activities of CCTs and SRC1 or SRC2 in MCF-7 cells.** (**A**) MCF-7 cells were co-transfected with the reporter plasmid pG5CAT (which expressed CAT), the pM construct of CCT (α, β, γ, δ, ε, ζ, η, or θ), and the pVP16 construct of SRC1. Control cells were transfected with only pG5CAT and the pVP16 construct of SRC1. CAT activity was measured at a wavelength of 415 nm. Error bars show the standard deviations (n = 6). (**B**) MCF-7 cells were co-transfected with the reporter plasmid pG5CAT (which expressed CAT), the pM construct of CCT (α, β, γ, δ, ε, ζ, η, or θ), and the pVP16 construct of SRC2. Control cells were transfected with only pG5CAT and the pVP16 construct of SRC2. CAT activity was measured at a wavelength of 415 nm. Error bars show the standard deviations (n = 6).
(TIF)

Figure S4 Effects of the overexpression and/or knock down of AIB1 and/or CCTζ overexpression on the proliferation, spreading area, and cell cycle of MCF-7 breast cancer cells grown on silicone substrates with E_Y_ = 10 kPa (** ***P*** **<0.01).** (**A**) Cell spreading area of control, siAIB1, siCCTζ, ovAIB1, ovCCTζ, siAIB1+ovCCTζ, and siCCTζ+ovAIB1 cells grown on silicone substrates with E_Y_ = 10 kPa:. **P<0.01 compared with other groups. (**B**) The growth curves of control, siAIB1, siCCTζ, ovAIB1, ovCCTζ, siAIB1+ovCCTζ, and siCCTζ+ovAIB1 cells grown on silicone substrates with E_Y_ = 10 kPa. **P<0.01 compared with other groups. G2/M (**C**) G0/G1 (**D**), and S phase (**E**) of the cell cycle in control, siAIB1, siCCTζ, ovAIB1, ovCCTζ, siAIB1+ovCCTζ, and siCCTζ+ovAIB1 cells grown on silicone substrates with E_Y_ = 10 kPa. **P<0.01 compared with siAIB1.
(TIF)
